This article has been retracted.

# DNA methylome profiling at single-base resolution through bisulfite sequencing of 5mC-immunoprecipitated DNA

**DOI:** 10.1186/s12896-017-0409-7

**Published:** 2018-02-06

**Authors:** Zhen Jia, Yueyi Shi, Lei Zhang, Yipeng Ren, Tong Wang, Lejun Xing, Baorong Zhang, Guolan Gao, Rongfa Bu

**Affiliations:** 1 Department of Obstetrics and Gynecology, Beijing Aviation General Hospital, Beijing, 100012 China; 2 Department of Stomatology, Chinese PLA General Hospital, Beijing, 100853 People’s Republic of China; 3 Medical School, Nankai University, No.94 Weijin Road, Tianjin, 300070 China; 4 Department of Stomatology, Beijing Aviation General Hospital, Beijing, 100012 People’s Republic of China

**Keywords:** DNA methylome, MB-seq, MRB-seq, Novel technology, Single-base resolution

## Abstract

**Background:**

Detection of DNA methylome at single-base resolution is a significant challenge but promises to shed considerable light on human disease etiology. Current technologies could not detect DNA methylation genome-wide at single-base resolution with small amount of sequencing data and could not avoid detecting the methylation of repetitive elements which are considered as “junk DNA”.

**Methods:**

In this study, we have developed a novel DNA methylome profiling technology named MB-seq with its ability to identify genome-wide 5mC and quantify DNA methylation levels by introduced an assistant adapter *Alu*I-linker This linker can be ligated to sonicated DNA and then be digested after the bisulfite treatment and amplification, which has no effect of MeDIP enrichment. Because many researchers are interested in investigating the methylation of functional regions such as promoters and gene bodies, we have also developed a novel alternative method named MRB-seq, which can be used to investigate the DNA methylation of functional regions by removing the repeats with Cot-1 DNA.

**Results:**

In this study, we have developed MB-seq, a novel DNA methylome profiling technology combining MeDIP-seq with bisulfite conversion, which can precisely detect the 5mC sites and determine their DNA methylation level at single-base resolution in a cost-effective way. In addition, we have developed a new alternative method, MRB-seq (MeDIP-repetitive elements removal-bisulfite sequencing), which interrogates 5mCs in functional regions by depleting nearly half of repeat fragments enriched by MeDIP. Comparing MB-seq and MRB-seq to whole-genome BS-seq using the same batch of DNA from YH peripheral blood mononuclear cells. We found that the sequencing data of MB-seq and MRB-seq almost reaches saturation after generating 7–8 Gbp data, whereas BS-seq requires about 100 Gbp data to achieve the same effect. In comparison to MeDIP-seq and BS-seq, MB-seq offers several key advantages, including single-base resolution, discriminating the methylated sites within a CpG and non-CpG pattern and overcoming the false positive of MeDIP-seq due to the non-specific binding of 5-methylcytidine antibody to genomic fragments.

**Conclusion:**

Our novel developed method MB-seq can accelerate the decoding process of DNA methylation mechanism in human diseases because it requires 7–8 Gbp data to measure human methylome with enough coverage and sequencing depth, affording it a direct and practical application in the study of multiple samples. In addition, we have also provided a novel alternative MRB-seq method, which removes most repetitive sequences and allows researchers to genome-wide characterize DNA methylation of functional regions.

**Electronic supplementary material:**

The online version of this article (10.1186/s12896-017-0409-7) contains supplementary material, which is available to authorized users.

## Background

DNA methylation is one of the most important aspects in epigenetic modification and it plays key roles in the regulation of gene expression. It predominantly occurs at the C5 position of cytosines (5mC) within CpG dinucleotides, but is also present at non-CpG cytosines (CHG and CHH where H = A, T, C) in embryonic stem cells in mammals and plants [1–3]. DNA methylation is involved in many biological processes including embryonic development, X chromosome inactivation, genomic imprinting and silencing of transposable elements [4, 5]. Aberrant DNA methylation is also unequivocally associated with the pathogenesis and progression of many diseases, including cancer and immunological dysfunction [4, 6]. Therefore, detection of 5mC sites and evaluating their DNA methylation levels are of great significance to understanding the relevance of DNA methylation patterns in diseases, which can greatly prompt the identification of new disease-related genes and potential drug targets [7].

Understanding the patterns of DNA methylation in normal and disease processes requires characterizing its status at the whole-genome level (methylome). Over the past few decades, bisulfite sequencing has emerged as the ‘gold standard’ technology for assessing DNA methylation and has been used widely as a targeted approach to investigate specific candidate regions of interest (ROIs) [8]. Bisulfite treatment of DNA followed by PCR amplification leads to the chemical conversion of unmethylated Cs to Ts while leaving methylated Cs unchanged. Combining this technique with next-generation sequencing – a recent advance in modern genomics that has developed at a pace that has outstripped Moore’s Law – is known as BS-seq and has proved to be the most powerful and complete strategy for the quantitative detection of 5mC at a single-base resolution [9–11]. However, BS-seq requires the sequencing of the entire genome and is prohibitively expensive for determining the DNA methylome of large genomes with large sample sizes. Therefore, it is quite impractical to employ the BS-seq to routinely investigate mammalian genomes and the epigenetic causes of complex diseases despite a continually falling cost per base of next-generation sequencing.

Within plants and mammals, however, the repertoire of 5mC only accounts for about 1–6% of total nucleotides of a given genome with the vast majority of 5mC occurring at CpG dinucleotides [7, 12]. In this respect, the application of BS-seq to decipher what amounts to a relatively small proportion of the genome is clearly an excessive approach. Currently, several methods have been developed to target 5mC and generate genome-wide landscapes of DNA methylation. Restriction enzyme-based methods, such as Reduced Representation Bisulfite Sequencing (RRBS) [13] and Methylation-sensitive Restriction Enzyme sequencing (MRE-seq) [14], combine genomic DNA digestion with certain restriction enzymes followed by high-throughput sequencing of digestion fragments. Both techniques offer single-CpG resolution but both build methylation maps that are concentrated around the distribution of enzyme recognition sites. Bisulfite padlock probes (BSPPs) capture sequencing [15] and array capture bisulfite sequencing [16] isolate ROIs for methylation profiling using probes or arrays, respectively. While both methods detect DNA methylation correctly and quantitatively, these hybridization-based methods are subject to several limitations, such as the interrogation of specific known sites and species, probe effects and cross hybridization. Methylated DNA immunoprecipitation sequencing (MeDIP-seq) and Methyl-Binding Domain sequencing (MBD-seq) capture the methylated fraction of genomic DNA with 5-methylcytosine-specific antibodies and MBD2 protein [17–19], respectively, and are followed by next-generation sequencing. While these techniques are less biased in global coverage than the aforementioned methods, they are most effective in the analysis of regions, rather than single base resolution, of high CpG content and methylation level.

In this study, we address the short-comings of the methods mentioned above and have developed a novel DNA methylome profiling technology we call MeDIP-bisulfite sequencing (MB-seq). MB-seq combines MeDIP-seq with conditional bisulfite conversion, and can detect individual 5mC sites precisely and determine their DNA methylation level at single-base resolution in a cost-effective manner. Furthermore, we have developed another novel but alternative method, MeDIP-repetitive elements removal and bisulfite sequencing (MRB-seq), which only interrogates 5mCs in functional regions through depleting repeat fragments after MeDIP enrichment.

## Results

### Characterization of MB-seq and MRB-seq

MeDIP-seq is well suited to characterizing the overall methylation level across a short region but not individual CpG sites [17, 20]. BS-seq on the other hand offers unprecedented breadth and depth of genomic coverage at single-base resolution; however, it is prohibitively expensive [10]. To overcome the shortcomings of MeDIP-seq and BS-seq, while taking the advantages of each, we modified the MeDIP-seq protocol to encompass the useful aspects of bisulfite sequencing so as to evaluate DNA methylation pattern at single-base resolution; Fig. 1a illustrates the basic workflow of MB-seq. As the methylated Illumina sequencing adapters would influence 5mC antibodies’ capture efficiency, an assistant adaptor named *Alu*I*-*linker (containing a methylated cytosine in *Alu*I recognition site) was introduced in MB-seq. Our results show that the *Alu*I linker with one modified methyl-site has no significant interference with the MeDIP enrichment (Additional file 1: Table S1). Briefly, the *Alu*I-linker is firstly ligated to sonicated DNA fragments followed by MeDIP capture and bisulfite treatment. Biotin-labeled *Alu*I*-*bisulfite primers are then used to amplify the ligated DNA fragments. To improve the effective sequencing reads, amplified PCR products are digested with *Alu*I enzyme and purified by streptavidin beads to remove digested *Alu*I linkers (Additional file 1: Table S2). Finally, purified DNA were ligated to Illumina paired-end sequencing adaptors and subjected to high-throughput sequencing.

**Fig. 1:** Schematic outline of the MB-seq and MRB-seq experiment. **a** Schematic drawing of MB-seq approach. Genomic DNA was randomly fragmented to 100–300 bp and ligated to *Alu*I-linkers with a methylated *Alu*I recognition site close to the T-overhang. The ligated-fragments were captured using methylcytosine antibody, then treated with sodium bisulfite and converted to double stranded DNA by amplification using biotin labelled *Alu*I primers. The *Alu*I-linker was digested and removed by streptavidin coupled beads. The linker-removed sequence was added 3’end A-tailing, then ligated to Illumina multiplexing adaptors following PCR amplification using Illumina paired-end PCR primers. The PCR products of 230–250 bases in length were size-selected on a gel and sequenced on the Illumina platform. **b** Schematic drawing of MRB-seq approach. Repetitive DNA elements were removed using Cot-1 DNA after MeDIP (based on the MB-seq approach). Cot-1 DNA was labelled with biotin and coupled with streptavidin, and the streptavidin-biotin-Cot-1 DNA was hybridized to enriched methylated DNA fragments via MeDIP to remove repeat fragments. The methylated fragments obtained (single/low copy DNA fragments) were then subjected to sodium bisulfite treatment, PCR amplification, *Alu*I digestion and sequencing library preparation, as per MB-seq

Previous studies have demonstrated that cytosine is heavily methylated in transposable elements and slightly methylated in CpG islands, which are frequently located in gene promoters or regulatory regions [21, 22]. It has been reported that approximately 50–60% of sequencing reads captured by methylation binding proteins or MeDIP antibodies are mapped to repetitive regions [23, 24]. As the biological function of repeat elements remains unclear, and these so called garbage genes will affect data output and diversity when doing bioinformatics analysis. Therefore, we developed a novel method based on MB-seq, called MRB-seq, which focuses on mapping 5mC in functional regions by removing repeat elements by beads conjugated with Cot-1 DNA after MeDIP enrichment (Fig. 1b). Briefly, the Cot-1 DNA was first labeled with biotin and coupled with streptavidin. Then, the streptavidin-biotin-Cot-1 DNA was hybridized to MeDIP products to remove repetitive fragments. Then the repeat-removed DNA fragments are processed following the MB-seq protocol.

### Data generation of MB-seq and MRB-seq

Previously, we have employed BS-seq to investigate the methylome of peripheral blood mononuclear cells (PBMCs) in a Chinese YH sample [21] . To ensure consistent data comparability, this study employed DNA from the same batch of YH PBMCs for MB-seq and MRB-seq that was used for the BS-seq study [21]. Initially, after trimming off adaptor sequences and removing low quality and clonal reads, 7.29 and 7.65 Gbp data was obtained for MB-seq and MRB-seq, respectively using the Illumina GAIIx sequencer. Table 1 display summary sequencing statistics for each method. For the 5.40 Gbp MB-seq data (74.12%) and 5.93 Gbp MRB-seq data (77.51%) aligned to the reference human genome, 4.60 Gbp (63.10%) and 5.19 Gbp (67.86%) was unique (exactly one location in the specific strand) for MB-seq and MRB-seq, respectively. We then evaluated the efficiency of bisulfite treatment by calculating the C to T conversion rate for all cytosines in CpH context (CpA, CpC or CpT dinucleotides) [21]. It was estimated that the bisulfite conversion rate of MB-seq and MRB-seq was at least 99.10% even if we assume that all 5mC in CpH dinucleotides were due to conversion failure, which maintains a false positive rate below 1%.

**Table 1:** General parameters of sequencing data for MB-seq and MRB-seq

	BS-seq*	MB-seq	MRB-seq	RRBS
Raw data (Gbp)	103.7	7.3	7.7	3.43
Mapped data (Gbp)	70.5	5.4	5.9	2.68
Mapped rate	67.9	74.1	77.5	78.1
Unique mapped data (Gbp)	64.4	4.6	5.2	2.58
Unique mapped rate	62.1	63.1	67.9	75.22
Conversion rate	99.7	99.3	99.1	99.6
Methylation level of C	3.1	7.22	6.9	3.5
Methylation level of CG	68.8	84.8	84.4	67.8
Methylation level of CHG	0.22	0.88	0.92	0.32
Methylation level of CHH	0.21	1.68	1.36	0.23
Total number of mCpGs identified	26,636,539	8,132,866	4,288,326	1,608,626

* The General parameters of sequencing data of BS-seq is obtained from the methylome of PBMCs in a Chinese YH sample [21]

Like previous studies [3, 21], we only included regions covered by at least three uniquely mapped reads to ensure accuracy in determining methylation status. Table 1 shows that in comparison with BS-seq we observe an increase in the proportion of 5mC identified by MB-seq and MRB-seq, which accounted for approximately 7.2% and 6.9% of all sequenced Cs (Table 1), respectively. Similarly, we also found a remarkable increase in 5mC in overall non-CpG sites (especially in the CHH context) in MB-seq and MRB-seq datasets. It is shown that only 0.21% of CHH had methylated sites in BS-seq, while increased to 1.68% and 1.36% in MB-seq and MRB-seq, respectively. The higher methylated percentage of 5mC in CG, CHG, and CHH contexts for MB-seq and MRB-seq compared with that of BS-seq reflected the considerable enrichment of methylated sites from MeDIP.

By comparing the MB-seq and BS-seq, we sought to determine if there was any significant bias in methylated CpG (mCpG) identification. Among the 26,636,539 mCpG identified in BS-seq (Table 1), 30.0% were covered by MB-seq at the sequencing depth used to determine methylation status (Additional file 1: Figure S1a). In fact, an additional 41.7% were also covered with methylated reads but were dropped from analysis due to the cutoff used to determine methylation status. Further investigation of the uncovered mCpG in MB-seq revealed that these regions exhibit low densities of CpG dinucleotides (Additional file 1: Figure S1b). Also, less sequence depth might be another reason for lower coverage compared with the BS-seq’s. Anyway, this observation indicates that MB-seq is theoretically able to identify the majority of methylated genomic regions that occur anywhere in the genome. Therefore, it could be a useful and flexible method for researchers in epigenomics field whom aim at whole genome methylation status evaluation in lower cost.

### False positive exclusion of MeDIP-seq by MB-seq

Actually, MeDIP-seq cannot be applied to identify individual 5mC sites in captured reads or distinguish un-methylated reads captured by 5mC antibody due to its non-specific binding; therefore, it significantly increases rate of false positive in detecting methylation levels. It is anticipated that the rate of false positive in MeDIP-seq may be reduced by encompassing bisulfite treatment in MB-seq. Our data from Fig. 2a revealed that methylation level increased with unchanged sequencing depth in MeDIP-seq. Such bias was more severe for lower methylation level regions though the depth of MeDIP-seq increases when methylation level is higher than 70%. Our observation was consistent with previous conclusion that MeDIP-seq were more sensitive to highly methylated, high-CpG densities [25]. This indicated that MeDIP-seq produced false positives information regardless of mCpG density and methylation level estimation was not accurate. In contrast, MB-seq produced a gradual increase in density of methylation sites with increased methylation level of individual sites measured by BS-seq (Fig. 2b), indicating that MB-seq was more accurate in quantifying the methylation level of a specific site or region by using density of 5mC instead of reads depth.

**Fig. 2:** False positive exclusion of MeDIP-seq by MB-seq. **a** The distribution of sequencing depth across different methylation levels in MB-seq. **b** The distribution of the density of methylation sites across different methylation levels in MB-seq. All information was obtained using a 200 bp window on the genome-wide level. **c** The distribution of read depth, density of methylation sites in MB-seq and methylation level of 5mC in BS-seq across a randomly genomic region. **d** Zooming in to a specific region, the red box shows a captured region with no methylated sites, which were nonspecific DNA fragments captured by 5’methylcytosine antibody. **e** The percentage of windows (200 bp) with less certain methylation sites

To further illustrate the precision of MB-seq, we randomly profiled a genomic region and annotated (1) MB-seq sequencing depth, (2) the density of methylated sites of MB-seq, (3) the methylation level of BS-seq and (4) CpG density. A trend revealed that increased CpG density was accompanied by a proportional increase in the methylaion level from BS-seq (Fig. 2c and Additional file 1: Figure S2a). This observation indicated that the density of methylated sites from MB-seq was associated with CpG density and the methylation levels of 5mC but not that of specific CpG sites. In assessing sequencing depth and density of methylated sites of MB-seq, we found that certain regions have been covered by reads with different sequencing depth but these regions were largely unmethylated based on BS-seq (Fig. 2d and Additional file 1: Figure S2b). These regions were most probably derived from non-specific binding of 5-methylcytidine antibody to DNA fragments, which was a previously observed caveat of MeDIP. Determining the false positive rate of MeDIP-seq is also not straight-forward because of varying sequencing depth and the occurrence of both methylated and unmethylated sites within the same captured reads. Using a 200-bp sliding window, we investigated the density of methylated sites across the whole genome (Fig. 2e). Among the 2,058,554 windows with enriched genomic fragments, it was shown that 5.01% had no methylated sites and 7.50% had only one methylated site. Taken three methylated sites as the cutoff for assessing methylation, we estimated that 14.0% of regions could be considered false positives.

### Less than one-tenth of sequencing data reach saturation for MB-seq and MRB-seq when compared with BS-seq

In comparison with BS-seq, MB-seq and MRB-seq as targeted bisulfite sequencing methods do not require the sequencing of an entire genome. To account for the cost-effectiveness of MB-seq and MRB-seq to measure the methylome, we plotted the percentage of covered CpG normalized to a single Gbp of sequencing data genome-wide (Fig. 3a). Obviously, MB-seq and MRB-seq had a significantly lower cost per CpG than BS-seq at a given sequencing depth. Between the two enrichment methods, MRB-seq was lower cost per CpG than MB-seq since its exclusion of repeat sequences.

**Fig. 3:** The genome-wide CpG coverage per Gbp and saturation analysis of BS-seq, MB-seq and MRB-seq. **a** CpG coverage per Gbp as a function of read coverage threshold for CpGs on the genome-wide level. Coverage of CpGs per Gbp was calculated as (CpGs covered with more than three reads)/all sequencing data in Gbp. **b** CpG coverage in different amount of sequencing data of BS-seq, MB-seq and MRB-seq

For any given sequencing-based methylation method, the question of how deeply to sequence a library remains moot, as it is directly related to balancing of the cost of a given coverage and resolution of methylation level. Since the majority of 5mC occurs in CpG dinucleotides, we assessed coverage in different amount of sequencing data to evaluate the saturation of sequencing depth. We found that the sequencing data of MB-seq and MRB-seq almost reaches saturation after generating 7–8 Gbp data (Fig. 3b, Additional file 1: S1c), whereas BS-seq requires about 100 Gbp data to achieve the same effect [1, 21]. Compared with RRBS, MB-seq and MRB-seq had a significantly higher CpG coverage (Fig. 3b) and mCpG coverage (Table 1) with twice sequencing data.

### Removal of repetitive DNA elements by MRB-seq

Figure 2a shows that for MB-seq, 8.3% of reads were located in coding regions, 0.2% in the 5’-UTR and 1.2% in the 3’-UTR, while the majority of reads were located in introns (34.8%) and transposons (48.7%). This percentage of reads in transposons is consistent with previous results derived from MeDIP-seq of normal human mammary epithelial cells (50%) and also BS-seq of YH PBMCs (51%). In light of this statistic, we developed MRB-seq by reducing the repeat fraction using Cot-1 DNA. Expectedly, Fig. 4a shows that the percentages of all investigated genomic features (except transposons) were increased in MRB-seq compared with MB-seq’s. And we could easily find that the percentage of reads in transposons (36.68%) was lower than that in MB-seq (48.72%), indicating that our repeat-removal strategy can successfully deplete repeat-containing sequences, which lead to a relative increase in coverage of other genomic features.

**Fig. 4:** Repetitive DNA elements depleting by MRB-seq. **a** Read disribution of MB-seq and MRB-seq across different genomic features. **b** Sequencing depth of MB-seq and MRB-seq across different genomic features. MRB-seq successfully depleted repeat sequences and increased the percentage of other genomic features. **c-e** Scatter plots displaying the correlation of methylation levels between MB-seq and MRB-seq in transposons (**c**), CGIs (d) and promoters (**e**). It is shown that, other than in transposons, the repeats-removal process did not significantly affect the methylation level of other genomic features

In terms of sequencing depth across different genomic features, Fig. 4b shows that the mean sequencing depth of transposons was decreased from 7.4× in MB-seq to 5.3× in MRB-seq. In contrast, fold coverage of all other regions was increased. Additionally, we also calculated the D-value distribution of reads number in different sequencing depth between MRB-seq and MB-seq (Additional file 1: Figure S3). There were more reads generated in MB-seq than in MRB-seq for transposons, whereas more reads were generated in MRB-seq for other genomic features. Based on a straightforward normalization of reads located in transposons with total sequenced reads, we estimate that the deleted repeat sequences in MRB-seq accounted for approximately 25% of the total reads and 50% of repeat sequences generated by MB-seq. Functional annotation of reads associated with repeat sequences between MB-seq and MRB-seq showed that the decreased repeat sequences in MRB-seq consist largely of SINEs and LINEs (data not shown).

Although Cot-1 DNA can remove repetitive elements [26, 27], its potential impact on methylation level estimation at different genomic features was not known. Therefore, we correlated methylation levels between MB-seq and MRB-seq for various genomic features (Fig. 4c-e). Whereas Pearson’s correlation for transposon elements was 0.33 between MB-seq and MRB-seq, all other genomics regions have a coefficient > 0.80 (Additional file 1: Figure S4). Of particular note, the correlations for promoters and CGIs were very high (*r* = 0.88 and 0.95, respectively). Given the highly concordance between MB-seq and MRB-seq for all regions other than transposons, the repeats-removal process does not significantly affect the methylation level at other genomic features.

### Quantification of DNA methylation level by MB-seq

Previous studies have indicated that methylation levels typically decrease at the 5′ ends of genes, particularly downstream of transcription start sites (TSS), which can suppress transcriptional initiation when methylated [1, 14]. Conversely, methylation levels are increased in the gene bodies of activated genes. Using a sliding window-based method [3, 10], we calculated the density of methylated sites of total CpG (Fig. 3a). Consistent with previous studies [21], MB-seq and MRB-seq also revealed the same pattern of DNA methylation of CpG profile as that of BS-seq, which showed a high DNA methylation level in gene body and distal promoter regions with a sharp shallow stepdown at the TSS (Fig. 5a and Additional file 1: Figure S5a). For non-CpG profile (Fig. 5b, c and Additional file 1: Figure S5b, c), a similar pattern was obtained from CHG/CHH methylation based on MB-seq and MRB-seq. In comparison with the non-CpG profile based on BS-seq, it was shown that the methylation level measured from TSS and gene bodies has increased in both MB-seq and MRB-seq because of the enrichment of methylated non-CpG fragments.

**Fig. 5:** The methylation levels of MB-seq and MRB-seq in gene-associated regions. **a** Average methylation level of CpG in gene-associated regions using MB-seq and MRB-seq. Gene structure is divided into seven different functional regions and shown on x-axis. The y-axis is the average density of methylation sites in a 200 bp window. The green vertical line shows the mean location of the transcription start sites (TSS). **b** Average methylation level of CHG in gene-associated regions from MB-seq and MRB-seq. **c** Average methylation level of CHH in gene-associated regions from MB-seq and MRB-seq. MB-seq and MRB-seq clearly reflect the pattern of methylation level across different functional regions because of the enrichment of methylated non-CpG fragments. **d** The concordance and difference of CpG sites between MB-seq and BS-seq. **e** On the genome-wide level, and **(f)** CpG island-only level, the CpG sites covered solely in the BS-seq dataset were derived from low methylation level

To further investigate the differences of methylation level between MB-seq and BS-seq, we assessed the concordance of CpG dinucleotides across the whole genome obtained by both methods (Fig. 5d-f). As expected, we found that there was a significant overlap between MB-seq and BS-seq, with 64.0% of CpGs covered by both methods. However, 33.72% and 2.24% CpGs were uniquely identified in BS-seq and MB-seq, respectively. We found that the majority (95.7%) of CpGs covered uniquely bythe BS-seq dataset presented low methylation levels, indicating that MeDIP preferred to capture highly methylated regions (Fig. 5e). The CpGs covered solely by MB-seq dataset were resulted from antibodies’ special affinity to some target sites. This would be useful to know more details about the YH methylome where not detected by BS-seq.

### Correction of the methylation levels determined by MB-seq

Another feature of MB-seq and MRB-seq is that they can be used to quantify methylation levels at single-base resolution. However, comparison of MB-seq and MRB-seq with BS-seq is not straight-forward because BS-seq measures the absolute methylation levels while the quantification from MB-seq and MRB-seq will be skewed somewhat due to the using of antibody to isolate methylated fraction of genomic DNA (Additional file 1: Figure S6).

Therefore, we developed a model to estimate the methylation level of CG within 100 bp windows among genome. First of all, we found that the depth of MB-seq had a similar profile with methylation of C on genome on YH bisulfate sequence (Fig. 2 C). And the coverage on of low-CpG promoter and CpG islands (CGI) had same trends on genome (Additional file 1: Figure S7). So we considered that site with a different depth in MB-seq methods was primarily aroused by the methylation level of total methylated cytosine (CG/CHH/CHG) (Fig. 6a, b). Furthermore, we found that the methylation level of total cytosine on genome had an elevated trend in MB-seq (Fig. 6c) because unmethylated fragments were not captured by the antibody and thus the methylation level was over-estimated compared to BS-seq. Therefore, with the depth of MB-seq and methylation level of cytosine which determined by MB-seq, we developed an algorithm to estimate the methylation of CG on an enriched region (see details in method). And we found that the CpG methylation level we estimated was consistent with BS-seq in low methylation level windows (methylation level < 40%), but the hyper-methylation levels (measured by BS-seq) windows on which the quantity of un-sequenced un-methylated fragments was usually overestimated in MB-seq by our algorithm and resulted in lower methylation level when compared with BS-seq, so a Δ was used to revised it. We established an algorithmic model by the genome-wide data to correct the relative methylation level to true methylation level and results showed that our model was reasonable and robust with Pearson value 0.86 compared with BS-seq directly (Fig. 6d).

**Fig. 6:** Revised CpG methylation level of MB-seq. **a** Depth within 1–10 X distributed with Methylation level of C on genome. **b** Distribution of depth within 0–2 X and methylation level of C on genome. **c** Difference of methylation level C between MB and BS in 200 bp windows (BS-MB). **d** Correlation between revised methylation level of CG in MB-seq and BS-seq in 200 bp windows on genomewide

## Discussion

An essential and key step in unraveling the complex roles of DNA methylation on phenotype is to generate high-resolution methylomes for given samples [7, 28]. However, this has been subject to technological constraints due to the lack of technologies offering a good balance between single-base resolution, high-throughput, cost and quantitative measurement of the DNA methylation level with scalability of sequencing depth and coverage [7, 9]. Originally in BS-seq, researchers ligated methylated sequencing adapters to sonicated DNA fragments and amplified to prepare a library for bisulfite sequencing [1, 21]. However, if MeDIP antibodies are used to capture the methylated genomic fragments, methylated sequencing adapter has effect on immunoprecipitation efficiency when it is ligated to sonicated DNA before MeDIP. And if bisulfite treatment is used prior to MeDIP enrichment, single stranded DNA cannot be ligated to methylated sequencing adapter. In this study, we have developed a novel DNA methylome profiling technology named MB-seq with its ability to identify genome-wide 5mC and quantify DNA methylation levels by introduced an assistant adapter *Alu*I-linker. This linker can be ligated to sonicated DNA and then be digested after the bisulfite treatment and amplification, which has no effect of MeDIP enrichment. In this way, we have successfully unified the two key steps between MeDIP and BS-seq to a novel method, namely MB-seq, to permit meaningful sequencing data, which can evaluate whole genome methylation profile at single-base resolution.

Among the currently available methods used to measure DNA methylome, undoubtedly, BS-seq provides a far more precise and comprehensive view of the methylome by combining single-base resolution, unbiased coverage, and absolute quantification of methylation level [9, 10]. Though next-generation sequencing technologies allowing the generation of sequence data on an unprecedented scale with remarkable reduction in sequencing cost [9], it is still quite impractical to employ BS-seq to routinely investigate mammalian genomes and the epigenetic causes of complex diseases. Based on previous studies, it was shown that about 90 Gbp of data has only an average sequencing depth of 15× per strand [1]. This problem is expanded when we bear in mind that within a multicellular organism, there are probably as many epigenomes as cell types – unlike genomic profiles, which remain generally identical regardless of cell type. Compared to BS-seq, MB-seq performed comparably well in terms of single-base resolution, 5mC identification and the quantification of DNA methylation level. On the other hand, we also could estimate the absolute methylation level of CG, especially in CG low methylation regions. An important advantage of MB-seq is its largely lower data requirements. We show that for MB-seq about 7–8 Gbp data could measure one methylome with enough coverage and sequencing depth, which is about 15 fold less than that of BS-seq, affording it a direct and practical application in the study of multiple samples.

Although 5mC predominantly occurs in CpG dinucleotides, recent genome-wide DNA methylation profiles have revealed that non-CpG methylation is a prevalent feature (25% of all 5mC) in human embryonic stem cells [1, 3]. Without enough sequencing depth, measuring the methylation level of non-CpG was not easy based on BS-seq, especially for the low methylation status of non-CpG and the effect of sequencing error. However, MB-seq could detect non-CpG methylation and also increase sequencing depth here due to the nature of enriching for methylated non-CpG sites. It was found that there were similar non-CpG profiles between BS-seq and MB-seq but with an increased methylation signals in the MB-seq dataset. Although the functional significance of non-CpG methylation has been suggested [1, 3], the detailed biological function in this type of epigenetic modification remains largely unclear. Increasing the signal of non-CpG methylation in our methods will be helpful to identify the low methylation level of CHH/CHG sites and the differentially methylated regions (DMRs) of non-CpG sites between samples, which could prompt our understanding of biological function of methylation in non-CpG sites.

In comparison to MeDIP-seq, MB-seq offered several key advantages. Firstly, due to bisulfite conversion, MB-seq is a single-base resolution method and can determine the location of 5mC precisely, unlike MeDIP-seq that merely reflects the methylation levels of a region dictated by library size selection [17, 20]. Second, due to single-base resolution, MB-seq can discriminate the 5mC within a CpG and non-CpG pattern. This capability along with above mentioned increased signal of non-CpG methylation will make MB-seq particularly attractive for the characterization of the methylome of given samples with abundant non-CpG methylation, such as human embryonic stem cells. Third, unlike MeDIP-seq, which is somewhat prone to potential false positive fragments due to non-specific binding of 5-methylcytidine antibody [17, 20], MB-seq can distinguish accurately between bona fide methylated sites and those captured fragments that show no evidence of methylated sites, which will permit a more precise quantification of methylation levels. Previous studies revealed that about 45% of the human genome consists of repeat elements and highly methylated DNA often presented in repeat-rich pericentromeric regions, such as transposable elements [22, 29]. Although DNA methylation in repetitive elements plays an important role in genomic stability, its function remains to be investigated. Because many researchers are interested in investigating the methylation of functional regions such as promoters and gene bodies, we have also developed a novel alternative method named MRB-seq, which can be used to investigate the DNA methylation of functional regions by removing the repeats with Cot-1 DNA. Cot-1 DNA has been widely used to block the hybridization of repeats presenting within DNA probes in a CGH microarray experiment or FISH assays [26, 27]. In this study, we showed that Cot-1 DNA can only remove ~50% of repeats (most of which are SINEs and LINEs), which indicates that it is difficult to remove repeat sequences via hybridization. Nevertheless, our result demonstrates that repeat sequences can be partially removed with no impact the methylation level of other genomic regions.

The accuracy of the DNA methylation levels derived from MB-seq and MRB-seq is accredited, suggesting that MB-seq and MRB-seq is a promising method for detection of methylomes in species with low global level of DNA methylation and plenty of repetitive regions, respectively. Whereas, the accuracy of BS-seq is generally dependent on sequencing depth. Consequently, BS-seq is costly to profile methylome on species with the low global DNA methylation level and abundant repetitive elements. Recently, MeDIP-Bseq provided the first unequivocal evidence of cytosine methylation in Drosophila, which has long been thought to lack cytosine methylation [30]. Therefore, we prospect that MB-seq could be implicated to detect methylomes for species such as Locusta migratoria, which have large genome with numerous repetitive elements but low CpG methylation levels. In summary, we offered a newly developed MB-seq method with powerful and cost-effective for DNA methylome profiling at single-base resolution. In addition, we have also provided a novel alternative MRB-seq method, which removes most repetitive sequences and allows researchers to genome-wide characterize DNA methylation of functional regions.

## Methods

### Sample preparation and MeDIP

DNA from YH’s peripheral blood mononuclear cells was extracted by QIAamp DNA Blood Mini Kit (QIAGEN). 10 μg of DNA was fragmented to a mean size of approximately 250 bp by a Bioruptor (Diagenode, Belgium), followed by the blunt polishing, dA addition to 3′-end, and *Alu*I linker ligation (Additional file 1: Table S3), according to the instructions of the manufacturer. Ligated products were purified with DNA Clean & Concentrator™-5 kits (ZYMO) and eluted in 1 × TE (10 mM TRIS-HCl, pH 8.0, 1 mM EDTA, pH 8.0).

Methylated DNA was pulled down by Weber et al.’s method with a few revisions [31]. Briefly, about 6 μg of sonicated DNA was denatured at 95 °C for 10 min and then placed on ice for 5 min. Immunoprecipitation was performed by incubating and rotating DNA at 4 °C overnight in 1 × IP buffer (20 mM sodium phosphate pH 7, 280 mM NaCl and 0.1% Triton X-100) and 10 μl of Anti-5-Methylcytosine (5mC) Antibody, clone EDL MC-4 (Monoclonal Antibody, MABE1081, EMD Millipore). 50 μl dynabeads (M-280 Sheep anti-mouse IgG – 6.7 × 10^8^ beads/ml, Invitrogen) pre-washed with 1% PBS-BSA buffer according to the manufacturer’s instructions, were added to the DNA-antibody mixtures with slow rotation and incubation at 4 °C for 2 h. The dynabead-Ab-DNA mixtures was then washed three times with 800 μl 1 × IP buffer and finally resuspended in 100 μl of proteinase K buffer (10 mM Tris-HCl pH 7.8, 5 mM EDTA and 0.5% SDS). 4 μl of proteinase K (50 mg/ml, Invitrogen) was added to the mixtures and incubated at 50 °C for 2 h with rotation. Enriched DNA was purified using Zymo Clean& concentrator-5 kit with 700 μl binding buffer according to the manufacturer’s instructions and re-suspended in 20 μl nuclease-free water. Purified DNA was detected by qPCR with SYBR to evaluate MeDIP recovery efficiency according to previous study and is shown in Additional file 1: Table S4.

### Repeated DNA removal

Repetitive sequences were removed according to Craig and Bolzer’s method with some modification [26, 27]. Briefly, biotin-labeled Cot-1 DNA was prepared by mixing 4 μl Cot-1 DNA (100 ng/μl, Invitrogen) with 5 μl 10 × Klenow buffer, 5 μl biotin/dNTP mix (0.35 mM biotin-16-dUTP, 0.65 mM dTTP, 1 mM dCTP, 10 mM dGTP, 1 mM dATP), 8 μl random primers (8 N, 1 μg/μl) and 3 μl Klenow Enzyme (exo-) (Fermentas) at 37 °C overnight. The resulted biotin-labeled DNA was cleaned up using QIAquick PCR purification kit according to the manufacturer’s instructions, and re-suspended in 20 μl EB. By pooling the products together from 4 such biotin-labeling reactions, a total of 5.2 μg biotin-labeled DNA was harvested.

The biotin-labeled DNA was then conjugated to streptavidin-dynabeads M-280. Briefly, 4 μg biotin-labeled DNA, dissolved into 100ul TE, was denatured at 95 °C for 10 min and placed on ice for 5 min. At the same time, 2 mg streptavidin magnetic particles (Invitrogen) were pre-washed according to the manufacturer’s instructions and re-suspended in 100 μl of 10 mM TRIS-HCl, pH 8.0, 1 mM EDTA, pH 8.0, 2 M NaCl (2 × binding and washing buffer). Then, 100 μl denatured biotin-labeled DNA was added to pre-washed streptavidin magnetic particles solution and incubated at room temperature for 30 min with axial rotation. The biotin-streptavidin mixture was then applied to a magnetic particle separator for 3 min and the supernatant was gently removed and discarded.

The streptavidin-dynabeads bound biotin-labeled Cot-1 DNA as a “subtractor” and dried MeDIP-enriched DNA as a “source” were re-dissolved in 100 μl 6 × SSC and 0.1% SDS, and hybridized at 65 °C overnight with axial rotation. When hybridized DNA was cooled to room temperature, tubes were then applied to a magnetic particle separator for 3 min and the supernatant was gently transferred to a new tube and purified using a MinElute PCR Purification Kit (Qiagen) following the manufacturer’s instructions, and re-suspended in 25 μl 1 × TE.

### Bisulfite treatment, PCR and linker digestion

DNA from MeDIP and MeDIP repeat-removal captures were treated with sodium bisulfite using the EZ DNA Methylation-Gold Kit (Zymo Research), respectively. Both bisulfite converted products were amplified for 10 cycles with 5-terminal biotin labeled *Alu*I primer (Additional file 1: Table S4) in 50 μl volume by mixing: 5 μl of 10× JumpStart buffer (Sigma); 0.5 μl JumpStart™ Taq DNA Polymerase; 1 μl of *Alu*I primer 1 (20 μM); 1 μl of *Alu*I primer 2 (20 μM); bisulfite-converted DNA (50–200 ng) and nuclease-free water under the following conditions: initial denaturation at 98 °C for 30 s; cycling was 98 °C for 10 s, 52 °C for 30 s, 72 °C for 30 s with 10 cycles; extension at 72 °C for 10 min.

300 ng of above PCR products were digested with 10 μl 10 × buffer 2 and 5 μl *Alu*I (10 U/μl, NEB) in the volume of 100 μl at 37 °C overnight to cut *Alu*I linker. Digested DNA was purified using QIA PCR Purification Kit and free *Alu*I linker in digested DNA was removed by streptavidin-dynabeads M-280. Briefly, 1 mg pre-washed streptavidin-dynabeads M-280 was resuspended in 100 μl 2 × B&W (Bind and wash) buffer, added to 100 μl of *Alu*I-digested biotin-labeled DNA resuspended in TE and incubated at room temperature for 30 min with axial rotation. The mixture was then applied to a magnetic particle separator for 3 min and the supernatant removed gently and purified using a MinElute PCR Purification Kit, and re-suspended in 25 μl 1 × TE.

### Library preparation and Illumina Solexa high-throughput sequencing

Sequencing libraries of purified DNA from *Alu*I digestion were constructed following the Illumina paired ends sequencing library protocol (Illumine, USA). Illumina multiplexing adapter1 (sequence 5′-pho-GATCGGAAGAGCACACGTCT-3′) and adapter2 (sequence 5′-ACACTCTTTCCCTACACGACGCTCTTCCGATCT-3′), in which all the Cs were un-methylated, were ligated to after A-tailing added the annealed DNA following the protocol of Illumina Solexa GAIIx. 150–250 bp inert size DNA bands were selected and purified, and then amplified with 10 cycles under JumpStart™ Taq DNA Polymerase’s reaction as above. 150–250 bp insert size DNA bands were purified and sequenced with Illumina GAIIx. The protocol to establish sequencing library for MRB is similar with the one of MB-seq.

### Bisulfite read alignment and methylation site identification

The alignment of bisulfite-treated short reads to reference YH genome was the same as our previous study. Briefly, the cytosines on the forward of short read (“original form”) were in silico replaced by thymines (“alignment form”) and the guanines on the reverse of short read were in silico replaced by adenosines. Meanwhile, each cytosine in genome sequences was converted to thymine (represents the plus strand) and each guanine in genome sequences was converted to adenosine (represents the minus strand). In total, four times’ reads aligned was carried using the SOAP software to get the best hit of a given pair-end short read [32]. Then, a straightforward seed-and-extension algorithm was employed for the alignment with 2 mismatches allowed in the seed (30 bp) and 5 mismatches in the whole read.

Methylcytosines were identified according to the criteria of YH methylome [21]. Briefly, each mapped read and the two strands of the YH genome were converted back to their original forms to generate an alignment between their original forms. Then, cytosines in the short read aligned to the corresponding cytosines in the plus strand of reference genome, or otherwise guanines in the short read aligned to the corresponding guanines in the minus strand of reference genome were considered to be potential 5mCs. To ensure the reliability of 5mCs identification, only bases with quality scores higher than 14 were considered for further analysis. The bisulfite conversion efficiency was calculated according to the C to T conversion rate for all cytosines in CpH context (CpA, CpC or CpT dinucleotides). The false positive rate of 5mCs identification was calculated as: *FP* %  = (1 − *r*) ∗ *N*_*CpG*_/*N*_*mCpG*_ ∗ 100%. Where *r* is the conversion rate of non-CpG dinucleotides, *N*_CpG_ is the total number of CpG dinucleotides, and *N*_mCpG_ is the total number of methylated CpG dinucleotides. The methylation level of a specific cytosine was calculated from the uniquely mapped reads. The methylation level of a specific CpG is calculated as the number of C-to-C matches divided by the sum of C-to-C matches and C-to-T mismatches.

To analyze the methylation characteristics in detail, we define terms that appear in the figures: we define one C-to-C (sequencing to reference) as a methylation group. In mammals, the density of methylation sites was defined by dividing the methyl group by CG number (where methylation mainly occurs at CpG sites) using a sliding window-based method in a 200 bp window. In other living organisms, the density of methylation sites is defined by dividing the methyl group by C number. We ensure a site’s methylation by using a binomial distribution and calculate the threshold when all C-to-C derived from unmethylated C do not convert to T in bisulfite processing.

### Algorithm for estimating DNA methylation level

We used the uniquely mapped reads to get the depth of each 100 bp windows among genome. Because density of methylation cytosine determined by MB-seq is highly linear with the true methylation level of C in YH cell lines (Fig. 2b), we used observed genome-wide methylation level of C (3.6%) to estimate methylation level of C in a window by:

1 $$ \kern2.25em {\mathrm{E}}_{\mathrm{c}}=\frac{{\mathrm{Depth}}_{\mathrm{i}}\times {\mathrm{methy}}_{\mathrm{average}}}{{\mathrm{Depth}}_{\mathrm{average}}}\kern0.75em \left({\mathrm{R}}_{\mathrm{mb}}-{\mathrm{E}}_{\mathrm{c}}<3.6\ \right)\kern1.75em $$

2 $$ \kern2.25em {\mathrm{E}}_{\mathrm{c}}={\mathrm{R}}_{\mathrm{mb}}-3.6\kern3.5em \left({\mathrm{R}}_{\mathrm{mb}}-{\mathrm{E}}_{\mathrm{c}}\ge 3.6\ \right)\kern1.75em $$

3 $$ \kern2.25em {\mathrm{R}}_{\mathrm{mb}}=\frac{{\mathrm{mC}}_{\mathrm{i}}}{{\mathrm{Depth}}_{\mathrm{i}}}\ast 100\kern8.25em $$

 Depth_i_was the total read depth on a 100 bp window, R_mb_ was the density of methylation cytosine determined by MB-seq. Then, we estimated the methylation level (E_c_) of C in a window based on the depth of MB-seq, and windows with huge depth on the sites of centromere were filtered out. On the other hand, reads may be obtained randomly in the hypomethylation regions. In order to get the methylation level more accurately, we only chose the enriched windows by Poisson *P* < 10e-5 in comparison of depth in a window with that of background within 5 k bps centered on the window. Then, we could estimate the methylation level of CpG as descripted below.

4 $$ \kern1em {\mathrm{R}}_{\mathrm{c}\mathrm{g}}=\frac{{\mathrm{R}}_{\mathrm{mb}}}{1+{\mathrm{D}}_{\mathrm{c}\mathrm{g}}\left(\frac{1}{{\mathrm{E}}_{\mathrm{c}}}-\frac{1}{{\mathrm{R}}_{\mathrm{mb}}}\right)}+\Delta $$

5 $$ \kern2.25em \Delta =\left\{\begin{array}{c}0\kern4em {\mathrm{R}}_{\mathrm{c}\mathrm{g}}\le 40\%\\ {}\frac{0.5\ast {\mathrm{R}}_{\mathrm{mb}}\ast {\mathrm{D}}_{\mathrm{c}\mathrm{g}}\left(\frac{1}{{\mathrm{E}}_{\mathrm{c}}}-\frac{1}{{\mathrm{R}}_{\mathrm{mb}}}\right)}{1+{\mathrm{D}}_{\mathrm{c}\mathrm{g}}\left(\frac{1}{{\mathrm{E}}_{\mathrm{c}}}-\frac{1}{{\mathrm{R}}_{\mathrm{mb}}}\right)}\kern1em {\mathrm{R}}_{\mathrm{c}\mathrm{g}}>\kern0.5em 40\%\kern0.5em \end{array}\right. $$

6 $$ {\mathrm{R}}_{\mathrm{mb}}=\frac{{\mathrm{mCG}}_{\mathrm{i}}}{{\mathrm{Depth}}_{\mathrm{i}}}\ast 100 $$

Where R_cg_ was the estimated methylation level of CpG in 100 bp window, R_mb_ was the density of mCpG in 100 window we tested, and D_cg_ was density of CpG in a window, which was calculated by total CG/total C in the window. While ∆ was the revised parameter for methylation level of CG.

## Conclusions

In this study, we have successfully unified the two key steps between MeDIP and BS-seq to a novel method, namely MB-seq, to permit meaningful sequencing data, which can evaluate whole genome methylation profile at single-base resolution. Because many researchers are interested in investigating the methylation of functional regions such as promoters and gene bodies, we have also developed a novel alternative method named MRB-seq, which can be used to investigate the DNA methylation of functional regions by removing the repeats with Cot-1 DNA. In this study, we showed that Cot-1 DNA can only remove ~50% of repeats (most of which are SINEs and LINEs), which indicates that it is difficult to remove repeat sequences via hybridization.

The accuracy of the DNA methylation levels derived from MB-seq and MRB-seq is accredited, suggesting that MB-seq and MRB-seq is a promising method for detection of methylomes in species with low global level of DNA methylation and plenty of repetitive regions, respectively. In summary, we offered a newly developed MB-seq method with powerful and cost-effective for DNA methylome profiling at single-base resolution. In addition, we have also provided a novel alternative MRB-seq method, which removes most repetitive sequences and allows researchers to genome-wide characterize DNA methylation of functional regions.

## Additional file

Additional file 1: **Table S1.** No adverse effect of methylated AluI-linker on MeDIP enrichment. **Table S2.** Evidence of a decreased percentage of sequenced AluI-linker following removal with streptavidin coupled beads. **Table S3.** AluI-linker sequences and primers used in this study. **Table S4.** The qPCR primers used to evaluate MeDIP recovery efficiency. **Figure S1.** Comparison of the concordance mCG sites identified from MB-seq and BS-seq. **Figure S2.** Example for the false positive exclusion of MeDIP-seq by MB-seq. **Figure S3.** The differences of read depth of each genomic feature between MB-seq and MRB-seq based on D-value distribution. **Figure S4.** Scatter plots showing the relationship between density of methyl groups in MB-Seq and MRB-seq for different genomic features. **Figure S5.** The methylation levels of BS-seq in gene-associated regions. **Figure S6.** Comparison of the methylation level differences between BS-seq, MB-seq and MRB-seq. **Figure S7.** Coverage of CGI and none-CGI promoter. (a) Coverage of each CGI distributed with methylation of C on genome. (b) Coverage of each none CGI promoter distributed with methylation of C on genome. (DOC 2899 kb)

## Abbreviation

MB-seq: MeDIP followed bisulfite sequencing
MRB-seq: MeDIP-repetitive elements removal-bisulfite sequencing
PBMC: peripheral blood mononuclear cells
YH: YanHuang (the name of first Asian genome project)
